# Study on 3D Clothing Color Application Based on Deep Learning-Enabled Macro-Micro Adversarial Network and Human Body Modeling

**DOI:** 10.1155/2021/9918175

**Published:** 2021-09-07

**Authors:** Jingmiao Liu, Yu Ren, Xiaotong Qin

**Affiliations:** ^1^General Graduate School of Keimyung University South Korea, Daegu 42601, Republic of Korea; ^2^School of Design, Sichuan Fine Arts Institute, Chongqing 401331, China; ^3^School of Art, Yanching Institute of Technology, Sanhe 065201, China

## Abstract

In real life, people's life gradually tends to be simple, so the convenience of online shopping makes more and more research begin to explore the convenience optimization of shopping, in which the fitting system is the research product. However, due to the immaturity of the virtual fitting system, there are a lot of problems, such as the expression of clothing color is not clear or deviation. In view of this, this paper proposes a 3D clothing color display model based on deep learning to support human modeling-driven. Firstly, the macro-micro adversarial network (MMAN) based on deep learning is used to analyze the original image, and then, the results are preprocessed. Finally, the 3D model with the original image color is constructed by using UV mapping. The experimental results show that the accuracy of the MMAN algorithm reaches 0.972, the established three-dimensional model is emotional enough, the expression of the clothing color is clear, and the difference between the color difference and the original image is within 0.01, and the subjective evaluation of volunteers is more than 90 points. The above results show that it is effective to use deep learning to build a 3D model with the original picture clothing color, which has great guiding significance for the research of character model modeling and simulation.

## 1. Introduction

With the continuous improvement of quality of life as well as the popularity of e-commerce, the fitting system to help people virtual fitting gradually comes into view. Shi et al. proposed a full-automatic 3D virtual assembly system based on the 2D whole body image and 3D garment model, constructed 3D human body model from 2D human body image input by users, and obtained that the system is stable and effective in simulation training [1]. Guo et al. proposed a remote fitting system for clothing e-commerce, which can simulate the body shape of consumers through physical assembly robot and help consumers realize remote fitting [2]. In order to solve the accuracy of body shape measurement in clothing fitting, Lu et al. proposed a synthetic dataset of human avatars under wide clothing, including 1500 synthetic people with different body shape, posture, clothing, skin color, and background [3]. Hu et al. led the team members to propose the first fully automatic general method for virtual fitting of clothing, hair, shoes, watches, necklaces, hats, and other items. A large number of experimental results show that this method can well realize dynamic fitting [4]. Liu et al. proposed a fitting method based on the 3D virtual assembly of human body contour, which only needs one RGB image and transfers garment texture to human body contour under the guidance of the UV texture map, and achieved good results in the test [5]. Kurniawati et al. proposed in 2020 to use Microsoft Kinect tracking technology and 3D modeling mixer manipulation technology to establish an interactive 3D virtual fitting room, and the system can evaluate the matching degree of clothing and help users choose the most suitable clothing [6]. According to the influence of COVID-19, Meng put forward a virtual garment fitting system for the convenience of consumers and studied the color saturation of the system. The experimental results show that the proposed method has high efficiency [7].

Based on the model parameters derived from inaccurate anthropomorphic data, Ziegler et al. proposed a comprehensive identification method for geometric parameters of the human lower limb kinematics model based on three-dimensional marker position and parameters for determining (cycling) gait trajectory [8]. Kimpara et al. proposed an active driving system based on the human body model with the cooperation of team members. The system adjusts the dynamics of the human body model so that the human body model can make a real response to the maneuver [9]. Han et al. proposed the sequence view of sequence tags as a new deep learning model based on RNNs' encoding and decoding structure. The results show that this method can more effectively aggregate sequence views to learn more distinctive global features [10]. Jiang et al. proposed an effective deep learning model based on the convolutional neural network, which was used for 3D underground mapping of 2D ground observation data to realize 3D address feature construction [11]. Chen and Huang have studied the feature extraction of the 3D art design model based on deep learning, proposed a 3D art network social communication method, and verified the feasibility of this method [12]. Zhang studied the application of the dominant color extraction algorithm in clothing image retrieval and proposed a main clothing image color feature extraction algorithm to extract the main colors in the clothing image [13]. Kim et al. proposed a digital transformation method of human clothing in the image, which combined the geometric and style characteristics of clothing with the neural network. Finally, in the virtual trial experiment, it showed better advantages than the traditional comprehensive method [14].

To sum up, at present, most of the research in the world is carried out on the construction and application of the human body model. In addition, with the improvement of demand, the research on the clothing color is also increasingly carried out. But it is not difficult to see that most of the research is superficial, by using the automatic drive of human modeling to simulate the transformation of clothing color, the generation of clothing color of virtual human character can be realized. This is the key to optimize the virtual simulation fitting system. Therefore, this research will combine the deep learning technology of artificial intelligence and use the human body modeling drive to study the generation of the two-dimensional clothing image to three-dimensional persona clothing color model. The convenient and effective method will have great value in theoretical research and practical application.

In this paper, the meanings for some important parameters have been explained in Table 1. With the help of this table, some equations can be understood easily.

## 2. Clothing Analysis Based on Deep Learning

### 2.1. Clothing Color Analysis

HSV color space is used in this study, which is composed of hue, saturation, and lightness. HSV color space is usually represented by the closed inverted cone, where *h* represents color information, i.e., hue, which means the spectral color position, *s* represents saturation, i.e., the proportion value between the selected color purity and the maximum purity of the color, and *V* represents brightness [15–17]. The top of HSV color space starts from red and goes counterclockwise. It is composed of red, yellow, green, cyan, blue, and magenta. Counterclockwise indicates hue. The change from the inside to the outside indicates the saturation of the color space, the inside represents 0, and the outermost represents 100% saturation. The change from bottom to top indicates the lightness. The color of the bottom point is black, and the lightness is 0. When it reaches the top, the lightness is 100%. Because the visual effect of color is affected by hue, saturation, and lightness, the color is adjusted according to the visual effect, as shown in Table 2.

As shown in Table 2, values are assigned in a counterclockwise direction, with red as 0°, yellow is 60°, green is 120°, Cyan is 180°, blue is 240°, magenta is 300°, and the value range of each color system is set to float up and down 30°. Saturation is the degree of purity of color. According to the information given in Figure 1, it is divided into 9 segments according to the saturation from inside to outside. Low saturation, medium saturation, and high saturation represent each of the three segments from inside to outside. In addition, the lightness represents the lightness of color. The lightness of color is divided into low lightness, medium lightness, and high lightness from bottom to top. The same HSV color space is divided into 9 segments from bottom to top, and the lightness occupies 3 segments from low to high, and the numerical range in the table is also divided equally according to this segmentation method.

### 2.2. Clothing Analysis of Pictures

Human body analysis is to segment the human image into multiple semantic blocks. It usually uses convolutional neural network architecture for feature recognition, and for the pixel loss caused by semantic inconsistency, it usually uses the conditional random field for subsequent processing. However, a large number of studies have found that the range of processing inconsistency of conditional random fields is very limited, and there may be poor marker graphs [18, 19]. Therefore, in view of the above problems, a new confrontational network is gradually emerging. The main reason is that the discriminator is introduced into the confrontational network to identify human parts, which can enforce a higher level of consistency [20, 21].

With the deepening of the research on the adversarial network, its shortcomings also begin to appear. For example, in the network model, only one adversarial loss is generated in the direction propagation of a single discriminator, and one adversarial loss trains the two target layers of local inconsistency and semantic inconsistency separately. And, the confrontational loss caused by a single discriminator will make the training imbalance, resulting in poor convergence of the model [22]. Therefore, the adversarial network used in this study is the macro-micro adversarial network (MMAN). The main feature of this adversarial network is that it contains two discriminators, which can identify the label images of different pixel sets. The framework of the 3D virtual model is shown in Figure 1.

As shown in Figure 1, the MMAN model framework is mainly composed of three parts, one of which is a dual output generator. For the input image, the model will automatically process the image size and then use the dual output generator to generate a low resolution tensor, from which the low-resolution and high-resolution label images can be obtained. The other is macrodiscriminator, which is composed of four convolution layers. Its main function is to monitor the low resolution output label image from the dual output generator so that the global semantic inconsistency will be punished. The third is the microdiscriminator, which has a shallow structure of three convolution layers. Its main function is to supervise the high-resolution tag map and punish the local inconsistency. The training process of the recognition model of the MMAN algorithm is analyzed. Firstly, given the figure image with the shape of 3*∗L∗W* and the tag image with the shape of *C∗L∗W*, the pixel classification loss can be expressed as follows:

(1) $$\begin{array}{c} L_{\text{mce}}\left(G\right)=\sum_{i=1}^{L\times W}\sum_{c=1}^{C}-y_{ic}\log\;{\hat{y}}_{ic}. \end{array}$$

In formula (1), it represents the double output generator, the number of background classes, and the authenticity probability of the first pixel in. When the first pixel is in, its value is 1. It represents the prediction probability of the *i*th pixel in *C*. When the *i*th pixel is in *C*, its value is 0. In order to ensure that the final output results of the dual output generator can maintain consistency and the loss value in the final image output is small, this study combines classification loss and adversarial loss to achieve consistency, so as to ensure the high quality of image output. See the following formula for the specific expression:

(2) $$\begin{array}{c} L_{\text{mix}}\left(G,D\right)=L_{\text{mce}}\left(G\right)+\lambda L_{\text{adver}}\left(G,D\right). \end{array}$$

In equation (2), *λ* is used to balance pixel classification loss and adversarial loss. *L*_adver_(*G*, *D*) is adversarial loss, which is*L*_adver_(*G*, *D*)=*E*_*x*,*y*_[log  *D*(*x*, *y*)]+*E*_*x*_[log(1 − *D*(*x*, *G*(*x*)))]. In addition, the combination mechanism of cross-entropy loss and antagonistic loss is used to supervise the top and bottom output of the dual output generator. The specific way is shown in the following equation:

(3) $$\begin{array}{c} L_{\text{MMAN}}\left(G,D_{\text{Ma}},D_{\text{Mi}}\right)=L_{\text{adver}}\left(G,D_{\text{Ma}}\right)+\lambda_{1}L_{\text{mcel}}\left(G\right)+\lambda_{2}L_{\text{adver}}\left(G,D_{\text{Mi}}\right)+\lambda_{3}L_{\text{mceh}}\left(G\right). \end{array}$$

In equation (3), *L*_mcel_(*G*) represents the cross-entropy loss between the output low-resolution label image and the small-size label image, *L*_mceh_(*G*) represents the cross-entropy loss between the output high-resolution label image and the original quality label image, *L*_adver_(*G*, *D*_Ma_) represents the confrontational loss of the output low-resolution label image, and *L*_adver_(*G*, *D*_Mi_) represents the confrontational loss of the output high-resolution label image. The purpose of the model is to control the relative importance of the four losses. The training tasks of MMAN are as follows:

(4) $$\begin{array}{c} G^{*},D_{\text{Ma}}^{*},D_{\text{Mi}}^{*}=\arg\underset{G}{\min}\underset{D_{\text{Ma}},D_{\text{Ma}}}{\max}L_{\text{MMAN}}\left(G,D_{\text{Ma}},D_{\text{Mi}}\right). \end{array}$$

*G*^*∗*^, *D*_Ma_^*∗*^,  and *D*_Mi_^*∗*^ in equation (4), respectively, represent the output of dual output generator, macrodiscriminator, and microdiscriminator after alternating optimization, and the final optimization result needs *L*_MMAN_(*G*, *D*_Ma_, *D*_Mi_) to converge.

## 3. 3D Virtual Model Clothing Color Generation

### 3.1. Selection and Pretreatment of Template Model

In this study, a framework of the clothing color system based on image three-dimensional persona is proposed, which is convenient to generate the virtual three-dimensional persona clothing model from the image quickly and conveniently. The framework of the model is shown in Figure 2.

As shown in Figure 2, the whole algorithm process is divided into three steps. First, the input task image is used for clothing recognition to realize the clothing analysis of the image. Then, the similar three-dimensional character model needs to be generated for the subsequent simulation operation, and the template model selection and preprocessing are carried out. The created 3D persona model is only a simple 3D structure, so in order to facilitate the clothing color adaptation of the model, it is necessary to expand the model by UV. The UV unfolding of the model is to realize the UV mapping of the three-dimensional model, which corresponds the surface position of the three-dimensional model to the position of the two-dimensional image, and then, the color filling of each pixel of the three-dimensional model can be realized, and finally, the color change of clothing can be presented on the three-dimensional model. For the expanded texture image, different bright colors are used to distinguish clothes and trousers, and the gray values of the two colors are stored in the model library. The sample model in the model library is processed accordingly, and the problem image with color differentiation is also obtained. At this time, the preprocessing of the model is completed.

### 3.2. Clothing Texture Color Feature Extraction

After realizing the region recognition of the coat and trousers, it is necessary to restore the clothing texture and color on the 3D model by using the relevant information in the picture. Firstly, the texture of the visible part of the clothing is mapped to the corresponding area of the 3D model according to the texture and color of the corresponding position of the image. In the process of image mapping, rotation operation is also needed to adjust the direction processing model, and the rotated image is adapted to the size value of the simulation image [23–25]. When the programming operation of image rotation is carried out, the reverse mapping method is adopted. The reverse mapping is the opposite of the mapping process, mainly through the coordinates obtained after rotation to reverse map the position coordinates in the image. The calculation method is shown in the following equation:

(5) $$\begin{array}{c} \left\{\begin{array}{c} y^{\prime }=y÷\;\cos\;\alpha -x^{\prime }*\;\tan\;\alpha ,\\ x^{\prime }=x÷\;\cos\;\alpha -y^{\prime }*\;\tan\;\alpha . \end{array}\right) \end{array}$$

In equation (5), the ordinate of the image mapping point obtained by reverse mapping and the abscissa of the position point obtained by mapping are represented by *y* and *x* and *α* represents the image rotation angle. The results are as follows:

(6) $$\begin{array}{c} \left\{\begin{array}{c} y^{\prime }=-x*\;\sin\;\alpha +y*\;\sin\;\alpha ,\\ x^{\prime }=x*\;\cos\;\alpha +y*\;\sin\;\alpha , \end{array}\right) \end{array}$$

(7) $$\begin{array}{c} \left\{\begin{array}{c} x=x^{\prime }*\;\cos\;\alpha -y^{\prime }*\;\sin\;\alpha ,\\ y=x^{\prime }*\;\sin\;\alpha +y^{\prime }*\;\cos\;\alpha . \end{array}\right) \end{array}$$

Equation (6) represents the coordinates of the calculated image after rotation, but it is generally believed that the origin of the image is in the upper left corner of the image. If this method is used to calculate the nonsquare image, there is a certain probability that a negative value will appear. Therefore, equation (7) is used for subsequent processing, the origin of the image is moved to the center of the image, and the coordinates in the original image are restored by equation (7). The calculation process is shown in the following equation:

(8) $$\begin{array}{c} \left\{\begin{array}{c} x-s\text{Wid}÷2=\left(x^{\prime }-\text{dWid}÷2\right)*\;\cos\;\alpha -\left(y^{\prime }-\text{dHgt}÷2\right)*\;\sin\;\alpha ,\\ y-s\text{Hgt}÷2=\left(x^{\prime }-\text{dWid}÷2\right)*\;\sin\;\alpha -\left(y^{\prime }-\text{dHgt}÷2\right)*\;\cos\;\alpha . \end{array}\right) \end{array}$$

In equation (8), *s*Wid represents the width of the original image, *s*Hgt represents the height of the original image, dWid represents the width of the image after rotation, and dHgt represents the height of the image after rotation. With the help of formula (8), the original image coordinates corresponding to the rotated coordinates are restored to facilitate the recognition of the pixels around the coordinates of the original image, and then, the relevant rules are used to process the pixel information. In order to ensure that the color value of each pixel exists, bilinear interpolation is used for processing, as shown in the following equation:

(9) $$\begin{array}{c} f\left(x,y\right)\approx \frac{f\left(Q_{11}\right)}{\left(x_{2}-x_{1}\right)\left(y_{2}-y_{1}\right)}\left(x_{2}-x\right)\left(y_{2}-y\right)+\frac{f\left(Q_{21}\right)}{\left(x_{2}-x_{1}\right)\left(y_{2}-y_{1}\right)}\left(x-x_{1}\right)\left(y_{2}-y\right)\\ +\frac{f\left(Q_{12}\right)}{\left(x_{2}-x_{1}\right)\left(y_{2}-y_{1}\right)}\left(x_{2}-x\right)\left(y-y_{1}\right)+\frac{f\left(Q_{22}\right)}{\left(x_{2}-x_{1}\right)\left(y_{2}-y_{1}\right)}\left(x-x_{1}\right)\left(y-y_{1}\right). \end{array}$$

In equation (9), the abscissa of the middle point of the image and the ordinate of the middle point of the image are represented. *Q*_11_, *Q*_21_, *Q*_12_, and *Q*_22_, respectively, represent the position coordinates around the middle point, which are (*x*_1_, *y*_1_), (*x*_2_, *y*_1_), (*x*_1_, *y*_2_), and (*x*_2_, *y*_2_). This study is to calculate in HSV color space, but there will also be problems such as clothing pattern interference and recognition error, so we need to carry out extreme value elimination operation to get brighter clothing color. For the elimination of the extreme value, first calculate the mean value of the three factor channel in HSV, see the following equation:

(10) $$\begin{array}{c} vH_{1}=\frac{\sum_{i=1}^{m}x_{Hi}}{n},\\ vS_{1}=\frac{\sum_{i=1}^{m}x_{Si}}{n},\\ vV_{1}=\frac{\sum_{i=1}^{m}x_{Vi}}{n}. \end{array}$$

In equation (10), *vH*_1_ represents the mean value of hue, *vS*_1_ is the mean value of saturation, and *vV*_1_ represents the average value of lightness, which is the three-channel value of the pixel in HSV color space, and then traverses all pixels through the following equation:

(11) $$\begin{array}{c} s_{x_{1}}={\left(vH_{1}-x_{Ri}\right)}^{2}+{\left(vS_{1}-x_{Gi}\right)}^{2}+{\left(vV_{1}-x_{Bi}\right)}^{2}. \end{array}$$

In equation (11), *s*_*x*_1__ represents the difference between each pixel and the mean value. After eliminating according to the extreme value, the value of the pixel will not appear too large, so as to ensure that the color value deviation of the pixel is reduced. Finally, the proposed method is used to construct the 3D virtual decision-making clothing model, and the generated model is color rendered.

## 4. Analysis of Experimental Results

### 4.1. Algorithm Performance Analysis

This paper analyzes the performance of automatic recognition of the MMAN algorithm. The experimental environment used in the experiment is a remote control server. The system is Linux system, and the GPU memory is 8 GB [26]. In addition, the deep learning framework construction and running environment is Cuda8.0, and the program is written with Python 3.7. The image database used in the experiment is LIP model library, and 20% of the model library is used as the test set, and 80% is used as the training set, and the first step is to train and test the deep learning model. The results are shown in Figure 3.

As can be seen from Figure 3, with the increase of the number of iterations, the accuracy of the model in the training set gradually improves, and when the number of iterations reaches 20, the accuracy reaches the maximum value, and the maximum value is 0.972, and then, with the increase of the number of iterations, the accuracy of the model almost remains unchanged. In addition, it can be seen that the loss rate of the model also shows a significant decrease with the increase of the number of iterations, and after the number of iterations reaches 30, the loss rate of the model drops to the lowest value and remains unchanged for a long time. After that, the convergence of the MMAN algorithm is analyzed in the experiment. Finally, the convergence of the algorithm is shown in Figure 4.

As shown in Figure 4, the convergence of the algorithm is good, in which the two parameters lossD-r and lossD-f represent the scalar value of the image in the generator pair discriminator, respectively. It can be seen that the values of the two parameters are approaching 0.5 with the increase of test time. LossG represents the scalar value of the image output by the generator. As can be seen from Figure 5, its value gradually approaches 0. The values of the three parameters show that the MMAN algorithm is a good adversarial network, which means that the image generated by the generator can be passed by the discriminator for subsequent operation.

### 4.2. Actual Application Effect of Virtual Model

The experimental environment is win7SP1 operating system, the host is Intel Corei7-2600 CPU, the system memory is 8 GB, the program running environment is visual studio 2013, and the OpenGL interface is used for the final model display and human-computer interaction. Firstly, the extreme value elimination used in the experiment is analyzed, and its advantages are discussed, as shown in Figure 5.

As shown in Figure 5, in the experiment, the results of clothing color style extraction under the average value are compared with those obtained after eliminating the extreme value. It is not difficult to see that the results of clothing color style obtained by the two methods after processing the input image are almost the same. However, it can be concluded from the final presentation effect that the extracted value of clothing color style after the elimination of the extreme value is brighter, and the color saturation has also been significantly improved. From the visual effect point of view, it is more suitable for human visual senses. Then, the color model of 3D virtual character clothing is constructed, and the results are shown in Figure 6.

Figures 6(a)∼(c) show the virtual three-dimensional role model established after extracting the clothing color from the male input image, and Figures 6(d)∼(f) show the virtual three-dimensional role model established after extracting the clothing color from the female input image. As can be seen from Figure 7, the final three-dimensional model is relatively clear whether it is for men or women, and it can be seen that the clothing color of the characters in the image is also more accurate in the model. At the same time, it is undeniable that the pattern color on the clothing can be clearly expressed, and the position coordinates on the model are almost similar to those in the original picture. In order to show the effect of the 3D virtual persona clothing color model more scientifically and objectively, this experiment also analyzes the color difference after the model is established through the regional division of the model position and the objective color error detection, as shown in Figure 7.

As shown in Figure 7, greater than 0 means the color is brighter, and less than 0 means the color is darker. The established male and female models are divided into 100 regions for color difference detection. It can be seen that the fluctuation of the clothing color curve in male and female 3D virtual models is small. By comparing with the original color, you can find that the color difference curve of the 3D model changes little in light and shade. The above results show that the three-dimensional virtual character clothing color model established in this experiment is more successful, which can clearly show the clothing color information in the original picture, so as to facilitate the user to carry out the later clothing virtual try-on.

The final effect of the model needs to be verified by case analysis. This study randomly invited volunteers of different grades from different universities. The reason is that the consumption level of college students on the Internet is relatively heavy. Through the investigation of college students, it can have strong persuasion. Considering that the establishment of the 3D human model will be affected by multiple characters in the picture information, only a single character picture is collected in this study. There are 115 volunteers in this experiment, including 51 males and 64 females. The content of the survey is model aesthetics, clothing color, visual effect, and degree of interest. The total score of all content evaluation is 100 points. The results are shown in Figure 8.

As shown in Figure 8, the average score of male volunteers on the beauty of the model established in the experiment is higher, reaching 98 points, and the score of female volunteers on the beauty of the model is also up to 95 points, but it can be seen that all volunteers have higher scores on the clothing color effect displayed in the model, reaching 98 points. In addition, it can be seen that all volunteers are more interested in the clothes displayed after the model is established, which indirectly increases the shopping enthusiasm of users and contributes to the development of the Internet.

## 5. Conclusion

With the continuous development of the Internet, people gradually tend to the convenient life brought by the Internet, so the fitting system for online clothing shopping appears in field of vision, but there are many problems in the immature virtual fitting system, such as clothing color interference. Therefore, this study proposes a three-dimensional virtual human model based on deep learning and presents the clothing color in the human model with the help of clothing color extraction technology. In the process of virtual modeling, firstly, we need to use deep learning technology to analyze the color of human clothing and confirm the coordinates of the texture color by the method of reverse mapping. In order to meet the visual effect of color, we also need to eliminate the extreme value to ensure the quality of color in the model. The final results show that the MMAN algorithm has high effectiveness, and the accuracy rate reaches 0.972. At the same time, in practical application, it can be concluded that the model has high definition, complete clothing color and pattern, and clear position. Through the scientific and objective evaluation of clothing color, it is concluded that the color difference between the clothing color in the model and the original image is always within 0.01. According to the results of the investigation and analysis, it also shows that the model proposed in the study is in line with the public aesthetic, and the display of clothing color can also attract a large number of users. To sum up, the 3D virtual character clothing color object expression model established by deep learning is effective, and the clothing color remains intact, which can provide users with good visual effect and facilitate users to make a satisfactory decision when making online clothing selection. In addition, the results of this study will promote the development of the fitting system and optimize quality of life to a certain extent.

## Figures and Tables

**Figure 1:** The framework of the 3D virtual model.

**Figure 2:** Virtual 3D model framework.

**Figure 3:** Model training results.

**Figure 4:** Convergence of the algorithm.

**Figure 5:** Extreme value elimination effect. (a) Men's clothing. (b) Women's clothing.

**Figure 6:** Model construction effect.

**Figure 7:** Color difference of model dress.

**Figure 8:** Volunteer scoring.

**Table 1:** Formula interpretation.

Parameters	Interpretation
*L*	Image length
*W*	Image width
*C*	Number of background classes
*G*	Dual output generator
*L*_mce_	Pixel classification loss
*y*_ic_	Probability
*L*_adver_	Antagonistic loss
*λ*	Equilibrium parameters
*D*	Discriminator
*L*_MMAN_	Macro-micro adversarial network output
*L*_mcel_	Cross-entropy loss of low resolution and small size images
*L*_mceh_	Cross-entropy loss of high resolution and original images
*G* ^*∗*^	Dual output generator output
*D*_Ma_^*∗*^	Macrodiscriminator output
*D*_Mi_^*∗*^	Microdiscriminator output
*x*, *y*	Mapped abscissa and ordinate
*α*	Image rotation angle
*s*Wid	Original image width
*s*Hgt	Original image height
dWid	Image width obtained by rotation
dHgt	Image height obtained by rotation
*Q*	Coordinates around the midpoint
*vH*_1_, *vS*_1_, and *vV*_1_	HSV three factor mean
*s*_*x*_1__	Difference between pixel and mean

**Table 2:** Color setting.

Index		Numerical range
Hue	Red	330°∼360° and 0∼30°
	Yellow	30°∼90°
	Green	90°∼150°
	Cyan	150°∼210°
	Blue	210°∼270°
	Fuchsin	270°∼330°

Saturation	Low saturation	0∼33%
	Medium saturation	34%∼66%
	High saturation	67%∼100%

Value	Low value	0∼33%
	Medium value	34%∼66%
	High value	67%∼100%

## Data Availability

The data used to support the findings of this study are available from the corresponding author upon request.
